# Clinical efficacy of radical nephrectomy versus nephron-sparing surgery on localized renal cell carcinoma

**DOI:** 10.1186/s40001-014-0058-4

**Published:** 2014-11-06

**Authors:** Wentao Li, Yanlei Cheng, Yi Cheng, Hui Ren, Na Han

**Affiliations:** Department of oncology, Tongji Hospital, Tongji Medical College, Huazhong University of Science and Technology, NO. 1095 Jiefang Avenue, Wuhan, Hubei 430030 China

**Keywords:** Meta-analysis, Nephron-sparing surgery, Radical nephrectomy, Renal cell carcinoma

## Abstract

**Background:**

The aim of the present study was to compare the clinical efficacy of radical nephrectomy (RN) with nephron-sparing surgery (NSS) in treating patients with localized renal cell carcinoma (RCC).

**Methods:**

The literature search was performed in PubMed, MEDLINE Springer, Elsevier Science Direct, Cochrane Library, and Google Scholar up to December 2012. The software Review Manager 5.1 and the STATA software package v.11.0 were used for analyses. The odds ratios (ORs) and its 95% confidence interval (95% CI) were calculated for comparison. Subgroup analyses were performed based on the tumor size of RCC.

**Results:**

In total, 10 studies with 10,174 RCC patients (7,050 treated with RN and 3,124 treated with NSS) were selected. The pooled estimate (OR = 1.58, 95% CI = 1.15–2.15, *P* = 0.004) showed a significantly lower rate of cancer-specific deaths in the patients treated with NSS compared to RN. However, no statistically significant differences were found in the rate of tumor recurrence (OR = 0.84, 95% CI = 0.67–1.06, *P* = 0.14) and complications (OR = 0.91, 95% CI = 0.51–1.63, *P* = 0.74) between the patients treated with NSS and RN. In addition, all the subgroup analyses presented consistent results with the overall analyses.

**Conclusions:**

NSS had no significantly different from RN in tumor recurrence and complications for localized RCC. However, the significantly lower rate of cancer-specific deaths supported the use of NSS not only for RCC with tumor size >4.0 cm but also for tumor sizes ≤4.0 cm compared with RN.

## Background

Renal cell carcinoma (RCC) is the third most common malignancy of the genitourinary system characterized by lack of early warning signs, protean clinical manifestations, and resistance to radiotherapy and chemotherapy [1]. RCC patients account for approximately 3% of the adults with malignancy and 90% to 95% of the patients with neoplasms arising from the kidney [2]. In spite of the rapid development of medical technology, RCC remains a difficult malignancy to treat because of its ability to spread asymptomatically and its inherent resistance to conventional chemotherapy [3].

Currently, the available treatments for RCC consist of partial and radical nephrectomy (RN) [4]. Since the publication of Robson’s study in 1969 [5], RN has been regarded as the gold standard to treat localized RCC [6]. However, nephron-sparing surgery (NSS) has been increasingly advocated in recent years and has challenged this concept [7]. The main advantage of NSS is that it can preserve renal function after the removal of renal tumors [8]. However, whether NSS is a better treatment than RN for RCC still remains controversial. A recently published article reported that NSS substantially reduced the incidence of moderate renal dysfunction when compared with RN [9]. Another study showed that NSS seemed to be significantly less effective than RN in terms of overall survival in the intention-to-treat population [10].

Thus, in order to find the appropriate treatment for the patients with localized RCC and provide much needed evidence for clinical practice, we conducted a meta-analysis to compare the clinical efficacy of RN with NSS in patients with localized RCC.

## Methods

### Search strategy

We searched several public databases including PubMed, MEDLINE, Springer, Elsevier Science Direct, Cochrane Library, and Google Scholar up to December 2012. The key words “radical nephrectomy”, “nephron-sparing surgery”, “partial nephrectomy”, “renal cell carcinoma”, “renal tumor”, and “study” or “trial” were used to retrieve the potentially relevant literature. Meanwhile, the references of all relevant articles retrieved from above database were searched for any additional studies.

### Inclusion and exclusion criteria

The inclusion criteria were: i) the participants were patients with localized RCC; ii) the investigations of the patients were conducted during cardio pulmonary resuscitation after cardiac arrest; iii) the studies were prospective, retrospective, or cross-sectional studies; iv) the patients were divided into two treatment groups according to type of surgery (RN and NSS groups); v) the clinical outcomes, such as cancer-specific death, tumor recurrence, or complications, were investigated. We excluded the studies by the following criteria: i) only one treatment was investigated in the studies; ii) the studies did not compare results between RN and NSS; iii) the studies were non-original articles such as conferences, reviews, or reports. In addition, in cases of duplicate publication, only the study containing the most complete data was included.

### Data extraction and quality assessment

Two investigators independently extracted and assessed the information with the standard protocol and contacted the authors of included studies to obtain further information. Discrepancies were resolved through discussion with our research team or by contacting the original investigators. The data extracted from each study included general information (first author’s name, year of publication, country), participant information (sample size, age and gender of the patients in each group, tumor stage and size of patients), study design, and outcomes. When no appropriate quality evaluation criteria were found, the study quality was assessed by investigating the study methods, sample size, and design.

### Statistical analysis

The meta-analysis was performed by using the software Review Manager 5.1 and the STATA software package v.11.0. The odds ratios (ORs) and its 95% confidence interval (95% CI) as summary statistics were calculated to assess the treatment efficacy. The heterogeneity among the studies was evaluated by testing Cochran’s Q-statistic [11] and I^2^ statistic [12] with *P* <0.10 or I^2^ > 50, respectively. The pooled estimates of ORs were obtained by using the DerSimonian and Laid method in the random effects model [13]. The significance of the pooled ORs was determined by the Z-test (*P* <0.05).

In addition, it has been reported that different tumor sizes in RCC are associated with the clinical outcomes of treatment [14]. Therefore, subgroup analyses were performed based on the tumor size of localized RCC. Meanwhile, in order to test the reliability of the results, the sensitivity analysis was performed by sequential omission of individual studies. The funnel plot and Egger’s test (*P* >0.05) were used to assess the publication bias of the included studies.

## Results

### Literature search

A total of 908 potentially relevant articles were identified by initial search. The selection process is shown in Figure 1. Following removal of duplicated studies, 248 studies were retained. Then by scanning the titles and abstracts, 172 obviously irrelevant articles were excluded. Finally, 10 studies met the inclusion criteria following exclusion of 30 studies that lacked the required data and 36 studies that did not report the comparison between RN and NSS.

**Figure 1:** **Flow diagram of screening studies.**

### Characteristics of included studies

A total of 10 eligible studies [6,15-23] comprising 10,174 RCC patients (7,050 patients treated by RN and 3,124 patients treated by NSS) were included in the meta-analysis. The characteristics of these studies are shown in Table 1. The included studies were published from 2000 to 2012. The follow-up duration of these studies ranged from 10 to 208 months. The tumor stage and size varied between the studies.

**Table 1:** **Characteristics of the included studies**

**Study**	**Year of publication**	**Pathological stage**	**Tumor size (cm)**	**Duration of follow-up (months)**	**RN group**			**NSS group**		
					**Sample size**	**Age (mean ± SD)**	**Male (%)**	**Sample size**	**Age (mean ± SD)**	**Male (%)**
Lau et al. [15]	2000	T1	3.3^a*^, 3.7^b*^	120	164	NA	NA	164	NA	NA
Shinohara et al. [19]	2000	T1, T2, T3	<4.0	12 to 131	51	59	37 (73)	15	61	13 (87)
Poulakis et al. [17]	2003	NP	6.9^a*^, 3.9^b*^	14 to 27	199	65.2 ± 11.0	121 (61)	158	62.6 ± 9.9	110 (70)
Patard et al. [16]	2004	T1	4.0^#^	10 to 208	1075	60.0 ± 12.4	692 (64)	379	59.7 ± 12.3	253 (67)
Becker et al. [6]	2006	T1, T2, T3	3.7^*^	66^*^	369	60.2	225 (61)	241	59.4	150 (62)
Mitchell et al. [18]	2006	T1, T2, T3	5.2^*^	44^#^	66	66.9	44 (67)	33	68.9	26 (79)
Van Poppel et al. [21]	2007	T0,T1,T2,T3	<4.0	60	273	NA	178 (65)	268	NA	178 (66)
Antonelli et al. [20]	2012	T1,T3	>4.0	25 to 85	2345	62.5	1505 (64)	1,266	60.1	881 (70)
Huang et al. [23]	2009	NP	<4.0	48^#^	2435	NA	1362 (56)	556	NA	351 (63)
Gratzke et al. [22]	2009	T1, T2, T3	NA	11 to 71	73	NA	46 (63)	44	60.7 ± 12.4	29 (66)

SD, Standard deviation; RN, Radical nephrectomy; NSS, Nephron-sparing surgery; ^*^, Mean; ^#^, Median; ^a^, RN group; ^b^, NSS group; NA, Not clear.

### The results of statistical analysis

Cancer-specific death was assessed in five of the included studies [6,16,19,20,23]. The test of heterogeneity indicated that there was no significant heterogeneity (I^2^ = 30.0%, *P* = 0.22) among these studies. The overall pooled estimate (OR = 1.58, 95% CI =1.15–2.14, *P* = 0.0004) showed that there was a lower cancer-specific death rate in the NSS group compared with the RN group (Figure 2A).

**Figure 2:** **Forest plots of cancer-specific death (A), tumor recurrence (B), and complications (C).**

A total of five included studies reported the tumor recurrence of the patients [15,16,18-20]. No significant heterogeneity (I^2^ = 0.0%, *P* = 0.43) was identified. The overall pooled estimate (OR = 0.84, 95% CI = 0.67–1.06, *P* = 0.14) demonstrated that no significant difference existed between the two groups (Figure 2B).

Six studies [15,17-19,21,22] assessed the patient complications. The test of heterogeneity indicated a significant heterogeneity (I^2^ = 71.0%, *P* <0.01) among these studies. The overall pooled estimate (OR = 0.91, 95% CI = 0.51–1.63, *P* =0.74) did not show a significant difference in postoperative complication rate between RN and NSS group (Figure 2C).

### Subgroup analyses

The results of the subgroup analyses by tumor size are shown in Table 2. For all the subgroup analyses, the results of each indicator were consistent with the overall analysis (tumor size ≤4.0 cm: cancer-specific death, OR =1.69, 95% CI = 1.22–2.35, *P* =0.002; tumor recurrence, OR = 0.83, 95% CI = 0.66–1.05, *P* =0.13; complications, OR = 1.10, 95% CI = 0.31–3.92, *P* =0.88; tumor size >4.0 cm: cancer-specific death, OR =1.36, 95% CI =1.01–1.85, *P* = 0.04; tumor recurrence, OR = 0.87, 95% CI = 0.36–2.11, *P* = 0.76; complications, OR = 0.71, 95% CI = 0.44–1.13, *P* = 0.15) indicated consistent results with the overall analysis. However, inconsistent results are shown in the heterogeneity test. The heterogeneity among studies was significant in the overall analysis of complications. However, no significant heterogeneity among the studies was found in the analysis of tumor size >4.0 cm for complications (I^2^ = 0.0%, *P* =0.88).

**Table 2:** **Statistical analysis results**

**Subgroup of tumor size**	**Sample size**		**No. of studies**	**Meta-analysis**		**Test of heterogeneity**		**Egger’s test**
	**Case**	**Control**		**OR (95% CI)**	***P*** **value**	***P*** **value**	**I** ^**2**^ **(%)**	***P*** **value**
Cancer-specific death								
Overall	6,275	2,457	5 [6,16,19,20,23]	1.58 (1.15 to 2.15)	0.004	0.22	30.0	0.27
≤4.0 cm	3,930	1,191	4 [6,16,19,23]	1.86 (1.11 to 3.13)	0.002	0.17	41	–
>4.0 cm	2,345	1,266	1 [20]	1.36 (1.01 to 1.85)	0.04	–	–	–
Tumor recurrence								
Overall	3,701	1,857	5 [15,16,18-20]	0.84 (0.67 to 1.06)	0.14	0.43	0.0	0.58
≤4.0 cm	1,290	558	3 [15,16,19]	0.67 (0.27 to 1.64)	0.38	0.16	45	–
>4.0 cm	2,411	1,299	2 [18,20]	0.87 (0.36 to 2.11)	0.76	0.68	0	–
Complications								
Overall	826	682	6 [15,17-19,21,22]	0.91 (0.51 to 1.63)	0.74	<0.01	71.0	0.76
≤4.0 cm	488	477	3 [15,19,21]	1.10 (0.31 to 3.92)	0.88	0.0004	87	–
>4.0 cm	265	191	2 [17,18]	0.71 (0.44 to 1.13)	0.15	0.88	0	–

### Sensitivity analysis and publication bias

No inconsistent results were observed in the sensitivity analysis compared with the overall analysis; therefore, the stability and reliability of the results in this study were proved. No evidence of publication bias was shown by the funnel plot (Figure 3) and Egger’s test (*P* >0.1, Table 2).

**Figure 3:** **Funnel plot of complications.**

## Discussion

RCC is the most common cancer of the kidney. Currently, there is controversy regarding the clinical efficacy of NSS and RN in treating RCC. Thus, we performed this meta-analysis to compare the clinical efficacy of NSS and RN. The results showed that NSS had a significantly lower cancer-specific death rate compared with RN for RCC patients although there was no significant difference in the rate of tumor recurrence and complications between the patients treated by NSS or RN.

Our results confirm that NSS treatment has a significantly lower cancer-specific death rate compared to RN for patients with localized RCC. Based on its characteristics, NSS can protect from renal function loss associated with the removal of the full renal unit, as is performed in RN [24]. Further, Bouliere et al. reported that NSS is superior to RN in preserving renal function outcome even when expanding NSS indications beyond the traditional 4 cm cut-off [25]. Thus, the survival of patients treated with NSS may be increased due to less kidney damage compared to RN. This may be the cause for the lower cancer-specific death rate of patients treated with NSS compared to that of RN. Thus, NSS should be supported for the treatment of RCC. Robert et al. [26] reported that elective NSS can be performed with equivalent direct hospital costs and length of stay when compared with patients undergoing radical nephrectomy for small solitary RCCs. Another article reported that nephron-sparing surgery was the standard of care for small RCC [27]. Thus, the comparison of efficacy between NSS and RN with regards to other indicators still requires further evaluation.

In addition, the subgroup analysis showed the consistent results with the overall analysis, suggesting that tumor size did not influence the results of this study. NSS can be applied not only for RCC with tumor sizes >4.0 cm but also for tumors ≤4.0 cm compared with RN. However, the heterogeneity test indicated that no significant heterogeneity among the studies was found in the analysis of tumor size >4.0 cm for complications, while significant heterogeneity was found in the analysis of tumor size ≤4.0 cm and in the overall analysis. Therefore, tumor size is one of the sources of heterogeneity. Nevertheless, further studies are needed to explore other sources of heterogeneity. Moreover, clinical efficacy of NSS has been proven to be highly associated with different tumor stages or grades of RCC. Fergany et al. [28] reported that cancer-specific death was significantly affected by tumor stage in patients treated with NSS. In this meta-analysis, the tumor stage was different in each study and therefore no appropriate grouping could be used for subgroup analysis. Hence, further studies should focus on the influence of different tumor stages on the clinical efficacy of NSS vs. RN.

Finally, some limitations of this study should be mentioned. First, only published studies were included in this meta-analysis; thus, the grey literature may be omitted. Second, significant heterogeneity among the included studies was found in the indicators of complication. The sources of heterogeneity need be explored in further studies. Third, only three indicators were used to assess the clinical efficacy of RN and NSS, other indicators should be considered in further studies. In addition, the included studies were not randomized controlled trials or case-control studies, and therefore the quality evaluation criteria of the studies were not determined. Thus, more studies need to be performed to verify the results of this meta-analysis.

## Conclusions

In conclusion, we compared the clinical efficacy of RN in treating localized RCC with NSS in this meta-analysis. The results showed that NSS treatment had a better clinical efficacy than RN for patients with localized RCC. However, more studies must be performed to verify the results of this meta-analysis.

## Abbreviations

95% CI: Confidence interval
NSS: Nephron-sparing surgery
ORs: Odds ratios
RCC: Renal cell carcinoma
RN: Radical nephrectomy
